# A Virtual Reality Algorithm for the Study of Clinical Efficacy of Sports Injury Rehabilitation Training

**DOI:** 10.1155/2021/6725625

**Published:** 2021-09-30

**Authors:** Yang Han

**Affiliations:** College of Humanities and Art, Henan Quality Polytechnic University, Pingdingshan, Henan 467000, China

## Abstract

This paper aims to explore the influence of virtual reality technology interactive rehabilitation training system and PT and OT operation therapy on the exercise function, daily life activity ability (ADL), and the quality of life in patients with a sports injury. In this context, this paper mainly designed three experiments to test the virtual rehabilitation system: two action experiments (experiment 1), two experiments with actions in 3 different positions (experiment 2), and five different actions (experiment 3), and the motion intention recognition rate, average total time, and task completion degree of the three experiments were calculated. The virtual scene and hardware equipment were kept stable, and the human-machine interaction effect was good. The effectiveness of the proposed virtual reality rehabilitation training system is demonstrated from other aspects. The results showed that the average completion time of 5 volunteers was 57.72 seconds, with an average offline accuracy of 89.03%. In experiment 2, the five volunteers averaged 54.98 seconds, with an average offline accuracy of 91.73%. The average recognition accuracy of the training system reached 90%, demonstrating the effectiveness of the virtual reality rehabilitation training system in terms of motor intention recognition rate, average total use time, and task completion.

## 1. Introduction

Virtual reality is interchangeable, which makes people have a complete sense of immersion. Another characteristic is imagination. The virtual image seen, the sound or music heard, and the environmental feedback can replicate the natural and virtual worlds with completely false illusions. So, the 3I characteristics of virtual reality technology are imaginative, immersive, and interactive. Virtual reality technology can also be applied in pharmacological studies. The researchers designed various virtual display simulators to simulate the action of drug molecules and biochemistry and observe the simulation results. This technique provides new methods for testing drug properties that can significantly accelerate the development of drugs to treat various diseases. At present, virtual reality rehabilitation technology in the medical field is applying virtual reality games to bring patients into the virtual reality game environment, simulating specific scenes, and adding force feedback and visual feedback technologies. This technology allows the patient to get immersive comfort in the rehabilitation training and avoids the dullness caused by repeated training. The application of virtual reality technology in the medical field is still in its infancy, but it has already had a significant impact on the medical field. Applying virtual reality technology to the clinical training of rehabilitation medicine, that is, through virtual reality environment, games, and other training modes, the patient is brought into a virtual reality environment similar to or completely unfamiliar with real life. By simulating specific daily life scenes such as open windows, pour water, and wipe tables, patients can cooperate with the robot for rehabilitation training during the game. These virtual scenes can be similar to the natural environment, such as the rehabilitation room, or a more friendly environment, such as the kitchen and bedroom of an ordinary family. The game design of virtual reality can easily guide patients to complete specific action tasks. Patients can practice safely alone, repeated training in specific movements, and enhanced neural reconstruction can significantly reduce the intensity of the treatment of the professional. The same doctor can also care for several patients simultaneously, significantly reducing labour costs and reducing the burden of the patient's family. In this process, the rehabilitation training robot collaborates with the virtual reality software program to collect the kinematics information of the patient, for example, parameters such as distance. Angle, angular velocity, acceleration, and force can reflect the rehabilitation training effect of patients and feedback to doctors to develop a more effective rehabilitation training program to analyze and evaluate the rehabilitation training effect of patients.

Three experiments were designed to test the virtual rehabilitation system. The virtual scene and hardware equipment remained stable during the experiment, and the human-computer interaction effect was good. The effectiveness of the virtual reality rehabilitation training system was proved from the aspects of intention recognition rate, average total time, task completion, etc.

In recent years, virtual reality technology has been widely used in the medical field. Virtual reality (VR) technology is a potential tool for cognitive process assessment and rehabilitation. Alashram et al. discussed the effect of virtual reality training intervention on TBI patients' cognitive function and discussed a compelling virtual reality treatment scheme [1]. Karami et al. provided a comprehensive meta-analysis to evaluate the effectiveness of VR in rehabilitation and training for patients with autism spectrum disorders [2]. Elsa et al. discussed the availability of a virtual reality-based protocol (“Rehabilitation Gaming System,” RGS) for AUD patients [3]. Under the background of the rapid development of modern information technology, medical colleges and universities in China have launched the innovation of education methods one after another and set off a wave of development and application of virtual reality technology teaching, which makes up for the deficiency of traditional teaching model. Duan et al. discussed the application of virtual reality technology in the teaching of balance function rehabilitation training, providing references and suggestions for applying virtual reality technology in the teaching of balance function rehabilitation training [4]. MJ et al. discussed the effect of virtual reality training on sitting posture balance in patients with spinal cord injury [5]. Bofanova et al. studied the application of virtual reality technology in prosthetic limb pain rehabilitation [6]. Fang et al. studied the application of virtual reality technology in the practical teaching of physical rehabilitation majors. The research method of virtual scene location mapping based on the virtual realization technology of upper limb rehabilitation training is adopted [7].

Virtual reality technology is also a potential tool for cognitive process assessment and rehabilitation. Virtual reality technology can intuitively provide a nearly natural cognitive rehabilitation training environment for patients with neuropsychological diseases. Tan et al. used virtual reality technology to construct specific and universal scenes related to MCI patients, restore and train patients' cognitive ability of scene memory, and help patients enhance or gradually restore their cognitive ability of scene memory. Virtual reality scenes with different contents such as life, environment, traffic, and tourism are constructed, and real-time detection is carried out by combining the EEG signals of patients in different scenes [8]. Virtual reality (VR) technology can effectively integrate cognitive and functional approaches into TBI rehabilitation. However, little is known about the effectiveness of virtual reality rehabilitation in treating cognitive impairments associated with traumatic brain injury. In response to these clinical and research gaps, Ettenhofer et al. developed NeuroDrive in a virtual environment, an intervention designed to improve cognitive performance, driving safety, and neurobehavioral symptoms. This preliminary clinical trial aims to investigate the feasibility and preliminary efficacy of neural drive technology in the rehabilitation of chronic brain injury [9].

Virtual reality is also a promising physical rehabilitation tool. Studies have shown that rehabilitation training supported by virtual reality is beneficial to task training, multisensory feedback, diversified rehabilitation tasks, and patients' enthusiasm [10]. Cai et al. outlined the application of immersive virtual reality assisted rehabilitation technology in stroke patients' gait rehabilitation and compared it with traditional rehabilitation methods [11].

In this context, the application of virtual reality technology to the clinical training of rehabilitation medical treatment, that is, through the virtual reality environment, games, and other training modes to bring patients into a virtual reality environment similar to real life or completely unfamiliar, three experiments were designed to test the virtual rehabilitation system. During the experiment, the virtual scene and hardware equipment remained stable, and the human-machine interaction effect was good. The effectiveness of the virtual reality rehabilitation training system was proved from the aspects of intention recognition rate, average total time, task completion, and so forth. It can be applied to rehabilitation training for patients with forearm amputation.

## 2. Research Methods

### 2.1. Data Acquisition

Virtual reality technology can also be applied in pharmacological studies. The researchers designed various virtual display simulators to simulate the action of drug molecules and biochemistry and observe the simulation results. This technique provides new methods for testing drug properties that can significantly accelerate the development of drugs to treat various diseases. The assessment of motor function mainly includes assessing muscle strength, muscle tension, and range of motion, but these aspects are difficult to test directly. In clinical practice, patients generally need to complete the related activities for evaluation.

Firstly, the training data required by the EMG classification model should be collected. There are three types of data:

1. The EMG signals of two movements were collected: the subjects were seated in the experimental chair, the collected arm was slightly raised, and the hand relaxation (NM) and fist-clenching (HC) movements were collected while holding a fixed position.
2. Collect EMG signals of 2 movements in 3 different positions: collect subjects sitting in experimental chairs, facing the computer screen, the collected hand is raised to the upper left, upper right, and middle of the screen, respectively, and the EMG signals of hand relaxation (NM) and clenched fist (HC) movements are collected.
3. Collect EMG signals of 5 different movements: the collection process of subjects is the same as that of A. Hand relaxation (NM), clenched fist (HC), carpal adduction (WF), wrist abduction (WE), and hand opening (HO) movements are collected, respectively, with the arm in a fixed position.

Then, the collected data were saved into TXT format files. A support vector machine carried out the training to calculate the offline classification accuracy and save the training model.

### 2.2. Experimental Method

**Experiment 1 .**

It is an experiment of two movements. The dichotomy training model was imported in the experiment, and mode 1 of the two-dimensional virtual scene was selected for the task. There are three different spheres on the screen, one on the top left, one on the top right, and one in the middle. Control the virtual hand to grab the virtual ball into the three-ball frame. After each ball is thrown into the frame, the count in the frame will increase, and the following virtual ball will randomly appear on the screen. The task of completing ten balls in a group is completed. Repeat three groups and calculate the average total time to complete the training task in real time. As shown in the figure, when the EMG signal gives the grasping command, the virtual hand grasps the virtual ball, and the virtual ball will change from red to yellow, indicating that the subjects have grabbed the ball. Then the virtual ball will be put into the ball frame through arm movement, and the count of the ball frame will be added by one, and the virtual ball will randomly appear in another place on the screen. At the same time, the timer in the interface also keeps recording the save time and the total time of each pitch in the TXT file until a set of pitches are completed.

Finally, the accuracy of the offline classification and the accuracy of real-time classification are calculated. Offline classification accuracy is achieved by collecting two segments of EMG signals from subjects, divided into training and test sets. After the model is trained, the test set with suitable labels is imported for feature extraction. Then the classification model is used for prediction and classification, and the predicted results are compared with the actual labels. The real-time classification accuracy is based on the subjects taking actions according to the experimenter's instructions and doing each action 40 times to judge whether the actions they have done are consistent with the real-time classification actions of the system. Finally, the real-time classification accuracy is counted.

**Experiment 2 .**

It is an experiment of movements in 3 different positions. The training model of six categories was imported, and the same training task was carried out as in Experiment 1. However, when calculating offline classification accuracy, since actions 1–3 are hand relaxation actions and 4–6 are hand clenching actions, the system only needs to determine whether the subject's current action is a relaxation action or a clenching action. Whether it is a relaxation movement or a squeezing movement and whether it is movements 1–3 or 4–6, as long as the judgment is accurate, also needs to be determined. In Experiment 3, there are 5 different movements. The training model of five classifications was introduced to calculate the real-time classification accuracy. Volunteers performed 200 actions according to the experimenter's instructions, and each action was performed 40 times. Finally, the number of correct and wrong times of real-time judgment was counted, and the accuracy of real-time classification was calculated.

**Experiment 3 .**

The experimental actions of Experiment 3 are fixed.

The experimental actions of the three experiments are shown in Table 1.

## 3. Results' Analysis and Discussion

Three experiments are designed: two actions, two actions in 3 different positions, and five different actions. Five healthy subjects were recruited to wear gloves to simulate forearm amputees, then collect muscle electrical signals from different hand movements and different arm positions, and finally participate in the designed virtual reality training task. Experiments 1 and Experiment 2 mainly verify the influence of different positions on the accuracy of EMG signal recognition. The experimental results are shown in Tables 2 and 3.

It can be seen from the table that the average total time spent under the same condition is different due to the different response abilities of different volunteers. In Experiment 1, 5 volunteers completed the task in 73 seconds, 53.2 seconds, 36.8 seconds, 43.6 seconds, and 82 seconds, respectively, with an average time of 57.72 seconds. The results are shown in Figure 1. The offline accuracy rates were 85.01%, 89.94%, 90.20%, 90.24%, and 89.78%, respectively, and the average offline accuracy was 89.03%, as shown in Figure 2.

In the second experiment, five volunteers completed the task in 63.5 seconds, 42.0 seconds, 60.1 seconds, 57.3 seconds, and 52 seconds, respectively, with an average time of 54.98 seconds; the results are shown in Figure 3. Offline accuracy rates were 95.07%, 91.42%, 88.36%, 92.05%, and 91.77% respectively, with an average offline accuracy of 91.73%, as shown in Figure 4.

The average time for subjects to complete the task was not significantly affected by directly classifying grasping and releasing movements into two categories or classifying the same movement in different positions in a more detailed way. The overall average time was faster than expected, mainly because the volunteers were all healthy people, and some experimental verification of amputees was still needed before the practical application. The recognition rates of both are about 90%, indicating that the virtual rehabilitation training system can effectively identify human EMG signals as the control source.

In this study, real-time test identification results of Experiment 2 and Experiment 5 were also statistically analyzed, as shown in Tables 4 and 5. In Experiment 1, the accuracy rates of 2 groups of 5 volunteers were 90.50% and 97.00%, respectively, and the average accuracy rate was 93.75%. It is shown in Figure 5. In the third experiment, the accuracy rates of 5 groups of 5 volunteers in the real-time test were 93.00%, 82.00%, 97.5%, 89.5%, and 94.00%, respectively, with an average accuracy of 91.2%, as shown in Figure 6.

These two tables can better reflect the actual situation that the system recognizes the subjects' movements in rehabilitation training. It can be seen from the table that the recognition rate of clenched fist movement in category 2 and category 5 is generally lower than that of other movements. Especially in classification 5, the main reason is that the related muscles used in fist clenching are similar to those used in other movements.

According to the experimental statistical results, the average recognition accuracy of the virtual training system for the subjects' movements has reached 90%, no matter it is two movement categories or five movement categories; it shows that the training system can be applied to the rehabilitation training of forearm amputation patients, and it has a specific practical value. However, the experiment designed in this subject only had five healthy subjects. The sample size was too small, and forearm amputees were not recruited for the training experiment, so there may be some deviation in the experimental effect of amputees. Therefore, further exploration and research are needed.

## 4. Conclusions

This paper tested the virtual rehabilitation system through three experiments. The virtual scene and hardware equipment are stable, and the human-machine interaction is good. The test results show that the effectiveness of the virtual reality rehabilitation training system is demonstrated in terms of motor intention recognition rate, average total time, and task completion and can be applied to rehabilitation training in patients with forearm amputation.

## Figures and Tables

**Figure 1:** The time taken by volunteers to complete the task.

**Figure 2:** Offline accuracy of volunteers' actions.

**Figure 3:** Time taken by volunteers to complete the task.

**Figure 4:** Offline accuracy of volunteers' actions.

**Figure 5:** Correctness rate of 2 groups of actions of 5 volunteers.

**Figure 6:** Correctness rate of 5 groups of actions of 5 volunteers.

**Table 1:** Three groups of experimental actions.

The sequence	Arm gesture	Action
Experiment 1	Fixed	Relax (NM)
		His fist (HC)

Experiment 2	The upper left	Relax (NM)
		His fist (HC)
	The upper right	Relax (NM)
		His fist (HC)
	In the middle	Relax (NM)
		His fist (HC)

Experiment 3	Fixed	Relax (NM)
		His fist (HC)
		Hands open (HO)
		Wrist outreach (WE)
		Arm adduction (WF)

**Table 2:** Average time and offline accuracy of Experiment 1.

2 classified subjects	Average total time (s)	Offline accuracy (%)
Volunteer 1	73.0	85.01
Volunteer 2	53.2	89.94
Volunteer 3	36.8	90.20
Volunteer 4	43.6	90.24
Volunteer 5	82.0	89.78

**Table 3:** Average time and offline accuracy of Experiment 2.

6 classified subjects	Average total time (s)	Offline accuracy (%)
Volunteer 1	63.5	95.07
Volunteer 2	42.0	91.42
Volunteer 3	60.1	88.36
Volunteer 4	57.3	92.05
Volunteer 5	52.0	91.77

**Table 4:** Experiment 1's real-time test identification results.

Action		Volunteers 1	Volunteers 2	Volunteers 3	Volunteers 4	Volunteers 5	Correct (%)
His fist	Correct	31	40	40	36	34	90.50
	Error	9	0	0	4	6	

Relax	Correct	36	40	40	40	38	97.00
	Error	4	0	0	0	2	

A combined	Correct	67	80	80	76	72	93.75
	Error	13	0	0	4	8	

**Table 5:** Real-time test identification results of Experiment 3.

Action		Volunteers 1	Volunteers 2	Volunteers 3	Volunteers 4	Volunteers 5	Correct (%)
Relax	Correct	36	35	40	40	35	93.00
	Error	4	5	0	0	5	

His fist	Correct	30	32	28	40	34	82.00
	Error	10	8	12	0	6	

Hands open	Correct	38	37	40	40	40	97.5
	Error	2	3	0	0	0	

Wrist outreach	Correct	38	33	40	32	36	89.5
	Error	2	7	0	8	4	

Arm adduction	Correct	38	39	36	40	35	94.00
	Error	2	1	4	0	5	

A combined	Correct	180	176	184	192	180	91.2
	Error	20	24	16	8	20	

## Data Availability

The data used to support the findings of this study are available from the corresponding author upon request.
